This article has been retracted.

# Comparative Study on the Effect of Various Aerobic Exercises on College Students' Weight Loss Based on Deep Learning Analysis

**DOI:** 10.1155/2022/6825919

**Published:** 2022-07-30

**Authors:** Fanghui Li, Yongtian Huang, Yijun Luo, Jing He

**Affiliations:** ^1^College of Physical Education, Pingxiang University, Pingxiang 337055, Jiangxi, China; ^2^College of Physical Education, Yichun University, Yichun 336000, Jiangxi, China

## Abstract

In order to solve the problem of higher obesity rate of college students and meet the needs of college students to lose weight effectively, a comparative study on the effect of various aerobic exercises on college students' weight loss based on in-depth learning analysis is proposed. The experiment shows that 30 subjects who voluntarily participated in the weight loss experiment and research were selected from a university, including 16 men and 14 women. It shows that aerobic exercise plays an important role in improving people's energy metabolism. Based on the deep unsupervised learning algorithm, this paper studies the effect of a variety of aerobic exercises on college students' weight loss. It is found that visceral fat obese people are easier to lose weight than outer skin fat obese people. With the help of aerobic exercise to lose weight, we should choose the aerobic exercise items significantly increased in EPOC during exercise recovery according to the obesity characteristics and types of different college students so that the effect of exercise weight loss is more effective.

## 1. Introduction

After entering the twenty-first century, with the continuous development of China's social economy, modern people's living standards have been greatly improved. At the same time, people's consumption habits and eating habits are undergoing great changes, and the impact of the improvement of living standards and the change in eating habits is also huge [1]. Obesity has even become the third major disease affecting human health in the twenty-first century after AIDS and cancer. Different degrees of obesity and other subhealth states affect people's health from different levels. In addition, the current eating habits and dietary structure are gradually developing towards high nutrition, high energy, and high fat. Under such living standards, people's health level has not improved with the improvement of living standards but shows a malignant development trend. More and more people are obese and begin to show a younger trend [2]. Even some young people have begun to cause a series of diseases such as tertiary education because of obesity. In other words, modern obesity has become an important factor affecting human life expectancy. A large number of experiments show that different types of aerobic exercise can effectively reduce obesity, improve people's immunity and physical quality, achieve different degrees of fat-burning effects through different intensities of aerobic exercise, and improve people's health levels while solving the phenomenon of obesity. Based on this, taking the deep learning algorithm as the starting point, a deep unsupervised learning algorithm is proposed. Through the comparison of the weight loss effects of different aerobic exercises, aerobic exercises that are more conducive to college students' weight loss are put forward [3].

From the above definition of deep learning, we can get: first, deep learning is a research subfield of machine learning (shown in Figure 1). Strictly speaking, the research on artificial intelligence includes game theory, machine learning, expert system, multiagent, and other technologies. Feature learning, which extracts some representative features from the original data, is a subdomain of machine learning; Deep learning of complex models is a subdomain of feature learning. That is, one of the tasks of deep learning is to extract appropriate features from the original data. Second, deep learning is a series of machine learning algorithms. Machine learning algorithms are divided into learning algorithms and unsupervised learning algorithms. Therefore, deep learning algorithms can also be divided into supervised deep learning algorithms and unsupervised deep learning algorithms. Third, deep research is multilevel nonlinear abstract data.

## 2. Literature Review

In 1943, Abrantes et al. and Zhu et al. established the first neural network calculation model MP model on the basis of combining mathematics and biology [4, 5]. In 1949, psychologist Bai et al. established the first rule of self-organizing learning, Hebbian learning, pointing out that when two neurons are excited at the same time, the strength of connection weight increases [6]. In 1954, Li first simulated the Hebbian network with a computer at MIT [7]. In 1958, Persiyanova-Dubrova et al. proposed the perceptron model 1% (perceptron model)—the well-known single-layer neural network model (the input layer is not included in the network layer measurement) is the first real artificial neural network model—and then proposed a two-layer neural network model with a hidden layer [8]. Zhang and Tian believe that aerobic exercise is the focus of many scholars' research and the most extensive method of weight loss [9]. Singh et al. have confirmed the effect and function of aerobic exercise on weight loss through a large number of studies [10]. Lee et al. in the research on the effect of aerobic exercise on weight loss, aerobic exercise, and aerobics have a good effect on women's weight loss. Through long-term aerobic exercise, we can effectively eliminate excess fat and reduce body weight. Among them, it has an increasing effect on fat volume, improving insulin, and controlling visceral fat content. By applying the neural network calculation model to exercise weight loss, we can effectively see the effect of weight loss [11]. At present, Darendeli and others have conducted in-depth research on the definition, classification, causes, harm, and weight loss methods of obesity, and many theories have been quite mature, which provides many useful references for us to grasp and define obesity scientifically in theory [12]. Although many experts and scholars have put forward different schemes and achieved certain results in the research on the intervention of aerobic exercise and resistance exercise on weight loss, they have verified the effect of aerobic exercise and resistance exercise on weight loss. However, the specific training intervention measures are too general, and the experimental data are not detailed enough. In particular, there are few research cases on the comparison of weight loss effects between aerobic exercise and resistance exercise. Most of them are limited to the analysis of fat reduction intervention effects of aerobic exercise combined with resistance exercise. There is a lack of research and evaluation on the effects and differences of different types of exercise, especially aerobic and resistance exercise on fat, body weight BMI, waist-hip ratio, cardiopulmonary function, and other sensitive indicators of obese people.

## 3. Method

### 3.1. Machine Learning and Human Brain Vision Mechanism

Machine learning is an interactive course that includes statistics, equation analysis, algorithm competition, theoretical theory, data theory, and other disciplines. It specializes in computer simulations of human behavior to acquire new knowledge and continuously researches and prepares existing knowledge to improve its performance [13]. Because a deep learning algorithm is a mechanism that simulates the visual information processing of the human brain, we will first discuss the definition of a learning algorithm in machine learning, then discuss the human brain visual mechanism, and then discuss the phenomenon of under- and overfitting in learning algorithm and two different learning types of supervised learning and unsupervised learning.

#### 3.1.1. Learning Algorithm

**Definition 1 .**

For some *T* function and measure function *P*, a computer is said to learn from knowledge *E* if it measures its performance in terms of P of *T* and improves with knowledge *E* [14]. For example, for the computer program of the man-machine game, the program obtains experience by playing chess with people. Its task is to participate in the man-machine game, and its performance is measured by the ability to win chess. In order to define a learning problem well, we must clarify three characteristics: the source of experience, the type of task, and the standard to measure the improvement of experience. Many learning problems can be defined in Figure 2, such as handwriting recognition learning involved in this paper and driverless learning by Baidu with a deep learning algorithm as shown in Figure 2.

#### 3.1.2. Human Visual Mechanism

The human visual system is the most amazing thing in the world [15]. The formation of large visual cues is scored in the visual cortex, as shown in Figure 3. The working process of the brain is an iterative and abstract process. After receiving the original data, the retina first receives information about the edge and direction by preprocessing area 1 and then receives information about contour and image. byThe additional abstractions of region 2, thus repeated by higher and higher abstractions, are always a more refined classification. Following the human brain's repetitive and problem-solving visual processing data from elementary to high level, a deep model has been developed [16]. Each layer of the depth network represents the area of the visual cortex, and the nodes on each layer of the depth network represent the neurons in the visual cortex. The information propagates from left to right, and the output of the lower layer is the input of the higher layer, which propagates iteratively layer by layer. From the definition of a learning algorithm, it can be seen that the main purpose of the deep network simulating the mechanism of the human brain's visual processing information is to store the experience of historical data in the network through the gradual learning of historical data, and the experience continues to improve with the increase of learning times.

It can be seen from the structure of the deep network that the input of high-level neurons comes from the output of low-level neurons without the interference of neurons in the same layer [17]. If the input layer is the feature representation of input data, it can be understood that the high-level features are the combination of low-level features, and the features from low-level to high-level represent the more and more abstract information processing process of the human visual system. An interesting problem is how to determine the size of the feature set, so as to effectively avoid under- and overfitting. If the size of the feature set is represented by capacity, the relationship between the feature set and training error and generalization error is shown in Figure 3. Increasing the number of feature sets reduces the training error, but the difference between the generalization error and the training error is increasing. When the difference between the generalization error and the training error is equal to the training error, the size of the feature is set as the visible error. When the difference between the generalization error and the training error is greater than the training error, the fitting function enters the overfitting state, and the fitting function is in the underfitting state between reaching the best feature set [18].

#### 3.1.3. Under- and Overfitting

Compared with the shallow network, the deep network established in Figure 4 has more parameters than the shallow network, which also means that for the feature set of the same size, the number of parameter unknowns of the deep network and the shallow network is different, which will lead to two problems of the impact of the size of the feature set on the deep network learning: The depth network is too small, resulting in its learning underfitting. The depth network is too large, resulting in its learning overfitting. For a clearer explanation, consider the single neuron model as shown in Figure 4, whose structure includes synapse, adder, and activation function [19].

When the activation function is linear transformation б(*x*) = *x*, a linear regression model is established. The regression vector formed by the input data with the number of features *n* is shown in the following formula:

(1) $$\begin{array}{c} X=\left[x_{1},x_{2},\ldots ,x_{n}\right], \end{array}$$

where *T* represents the transpose of the matrix. The output of neurons is represented by *α*, which constitutes the corresponding response. Because a single neuron has only a single output, *α* is a scalar. The input signal *x* on the synapse linked to the neuron is multiplied by the synapse weight *W* to obtain a linear regression model, and the parameterization is shown in the following formula:

(2) $$\begin{array}{c} \alpha =\sum_{i=1}^{n}w_{i}x_{i}+b, \end{array}$$

where *b* is offset. Using matrix notation, the compact form of formula (2) is as follows:

(3) $$\begin{array}{c} \alpha =W^{T}X+b, \end{array}$$

where *W* is the parameter vector, and the definition is shown in the following formula:

(4) $$\begin{array}{c} W=\left[w_{1},w_{2},\ldots ,w_{n}\right]. \end{array}$$

For a series of historical data, that is, training data, the task *T* of the learning algorithm is to calculate the parameters *W* and *b* through these training data. The experience *E* of the learning algorithm is to continuously improve the quality of parameters *W* and *b* so that it can accurately obtain the correct experience of historical data. The definition of training data is as follows:

**Definition 2 .**

A series of data pairs are as follows, as shown in the following formula:

(5) $$\begin{array}{c} \left(x^{j},y^{j}\right)\left(j=1,2,\ldots ,M\right). \end{array}$$

Input data formula and expected output data formula are as follows, respectively:

(6) $$\begin{array}{c} x\in R^{N_{1}}, \end{array}$$

(7) $$\begin{array}{c} y\in R^{N_{2}}. \end{array}$$

Define a performance measure *P* with the mean square error loss function *C*, as follows:

(8) $$\begin{array}{c} C=\frac{1}{2M}{\sum_{j}\left(y^{j}-a^{j}\right)}^{2}=\frac{1}{2}E\left[{\left\|Y-A\right\|}^{2}\right], \end{array}$$

where *M* is the number of training data pairs, *Y* is the expected output data vector, and *a* is the output vector of training data *x* through neurons. Equation (8) clearly shows that when the loss function *C* ≥ 0 and *a* approaches *Y*, *C* ⟶ 0. In addition to the mean square error, the loss function can also be expressed as mutual trust entropy, as shown in the following formula:

(9) $$\begin{array}{c} C=-\frac{1}{M}\sum_{j}\left[y^{j}1\text{n}\left(a^{j}\right)+\left(1-y^{j}\right)1\text{n}\left(1-a^{j}\right)\right]. \end{array}$$

Use formulas (2) and (3) to fit the function *f*(*x*) = *x*^2^ + *ε*, in which the odd points are used as the training data subset and the even points are used as the test data subset and use the model obtained from the training data subset to predict the values of the next 20 integer points. With the increase of *x*, the error increases accordingly as shown in Figures 5 and 6.

The reason for the poor generalization ability of this model is lack of fitting, that is, too small feature set makes the model too simple to reflect the real situation of the real model. When the feature set is too small, it is called underfitting. In this example, we use the linear regression function to fit the quadratic polynomial function, resulting in the linear function cannot fully reflect the characteristics of the original data set so that the generalization ability of the model for some newly added and unknown data is very poor, and finally, the learning algorithm fails [20]. For the underfitting caused by too small feature set, a natural solution is to increase the number of feature sets and construct a more complex model. The linear function is replaced by a higher-order polynomial function, but with the force increasing port of the number of feature sets, the number of parameters also increases, and the complexity of the model and the difficulty of solving the learning algorithm also increase accordingly. At the same time, it may also cause an overfitting phenomenon and lead to the learning failure of the learning algorithm.

According to the above idea, use the more complex cubic polynomial model instead of the simple linear model to observe the results as shown in the following formula:

(10) $$\begin{array}{c} f\left(x\right)=w_{1}x^{3}+w_{2}x^{2}+w_{3}x+b. \end{array}$$

Similarly, take the integer of the data set *x*∈ [0, 20], in which the odd points are used as the training data subset and the even points are used as the test data subset. The model obtained from the training data subset is used to predict the next 20 integer points, and the results are shown in Figure 7.

It can be seen from Figure 7 that with the increase in the number of parameters (number of feature sets), the error of cubic polynomial is smaller than that of linear function on the test data set, and its absolute error sum is also smaller than that of a linear function, which shows that the fitting accuracy of a cubic polynomial is better.

### 3.2. In-Depth Supervised Learning Model

#### 3.2.1. Model Building

Deep network model architecture composed of single neurons:

Assuming that the number of layers of neurons is *l* and the depth network is generally greater than 7, the *j*-th neuron of layer *L* is shown in the following formula:

(11) $$\begin{array}{c} \alpha_{j}^{l}=\sigma \left(\sum_{k}w_{jk}^{l}\alpha_{k}^{l-1}+b_{j}^{l}\right), \end{array}$$

where *w*_*jk*_^*l*^ is the weight value from the *k*-th neuron in layer *l*−1 to the *j*-th neuron in layer *l*, б is the activation function, and the S-type activation function is shown in the following formula:

(12) $$\begin{array}{c} \sigma \left(z\right)=\frac{1}{1+e^{-z}}. \end{array}$$

The function of activation is to obtain the summation node, as shown in the following formula:

(13) $$\begin{array}{c} z_{j}^{l}=\sum_{k}w_{jk}^{l}\alpha_{k}^{l-1}+b_{j}^{l}. \end{array}$$

After the nonlinear change, the neuron summation function is expressed in the input vector matrix, as shown in the following formula:

(14) $$\begin{array}{c} \left[\begin{array}{c} z_{1}^{l}\\ z_{2}^{l}\\ \ldots \\ z_{J}^{l} \end{array}\right]=\left[\begin{array}{c} b_{1}^{l},W_{11}^{l},\ldots ,W_{1\text{k}}^{l}\\ b_{1}^{l},W_{11}^{l},\ldots ,W_{1\text{k}}^{l}\\ \ldots \\ b_{j}^{l},W_{j1}^{l},\ldots ,W_{j\text{k}}^{l} \end{array}\right]\left[\begin{array}{c} 1\\ \alpha_{1}^{l-1}\\ \ldots \\ \alpha_{\text{K}}^{l-1} \end{array}\right]=\left[b^{1},W^{1}\right]\left[\begin{array}{c} 1\\ \alpha^{l-1} \end{array}\right]. \end{array}$$

According to the changed matrix, the output vector of layer *L* is nonlinearly transformed through the neuron activation function, as shown in the following formula:

(15) $$\begin{array}{c} \alpha^{L}=\sigma \left(z^{L}\right)=\sigma \left(w^{L}\alpha^{L-1}\right). \end{array}$$

Because the random gradient descent algorithm has a small amount of calculation when the training sample data is large, its calculation speed is fast. Therefore, when using a gradient descent algorithm to solve the minimum optimization problem with large training data set, the random gradient descent algorithm has a better effect than the batch gradient descent algorithm. Compared with the batch gradient descent algorithm, the convergence speed of each iteration of the random gradient descent algorithm is generally not as fast as that of the batch gradient descent algorithm, and the final iterative result of the random gradient descent algorithm is only hovering near the optimal solution calculated by the batch gradient descent algorithm. However, the time complexity of each calculation is smaller than that of the batch gradient descent algorithm. It is suitable for the situation of large-scale training data and low accuracy requirements.

To sum up, the parameter learning process of a deep network is divided into two steps: the first step is feature learning, that is, the bottom-up unsupervised layer-by-layer greedy training algorithm is adopted. First, a single-layer network is constructed. Each layer adopts the self-coding algorithm for parameter learning, adjusting one layer at a time, adjusting layer by layer, and finally obtaining the feature a priori information of unlabeled data. The second step is to fine-tune the whole network parameters, that is, adopt top-down supervised learning; add a classifier at the top of the network based on the parameters of each layer obtained in the first step; and then fine-tune the whole network parameters through a small amount of supervised learning with labeled data [21, 22].

## 4. Results and Analysis

Thirty subjects who volunteered to participate in the weight loss experiment and research were selected from a university, including 16 men and 14 women [23]. Depending on advertising and execution, the number of courses in the next step will increase further. The main data of the research project are shown in Table 1.

In order to effectively observe and compare the implementation and grouping of the experiment, the subjects were divided into the aerobic training group (*n* = 15: male 8, female 7) and resistance training group (*n* = 15: male 8, female 7) after further adjusting gender, age, body fat level, and physical strength level according to individual differences on the basis of fully considering the willingness of subjects to exercise and lose weight. The aerobic training group took the prescription for aerobic exercise and the resistance training group took the prescription for resistance exercise [24].

The subjects were trained and tested in groups, and the three fixed principles were adopted, that is, the test time, testers, and test instruments were fixed and the same, and the test cycle was set as 8 weeks. All participants were required to strictly follow the implementation requirements and execution of the exercise prescription formulated in this study [25]. At the same time, in order to avoid other relevant factors interfering with the exercise training and the final experimental results, relevant living and dietary requirements are put forward for all Table 2 experimental subjects. It is suggested that the experimental subjects should have a reasonable diet, control tobacco, and alcohol and avoid overeating during the test Table 3 cycle. In terms of daily work and rest, it is suggested to have a scientific regular work and rest, go to bed early, and get up early. At the same time, during exercise, pay attention to Table 4 supplement water and reasonably select relevant safe exercise protective equipment.

1. Compare the previous body composition test results, as shown in Table 2.
2. Table 2 shows that there is no significant difference between the aerobic exercise group and the resistance exercise group in body weight, BMI, body fat (%), lean body weight, waist-hip ratio, and other indicators before the formal intervention, *P* > 0.05, indicating that the body composition of aerobic exercise group and resistance exercise group is basically the same, which meets the experimental requirements and conditions as shown in Table 3.
3. According to Table 3, the aerobic exercise group and the work group had no significant difference in the ability and cardiac function before the intervention, *P* > 0.05, indicating that the difference in cardiac function was not statistically significant. Before the intervention of the two groups, it was suitable for the needs of the experimental operation [26] as shown in Table 4.
4. Before the intervention, there was no significant difference in body mass index, cardiopulmonary function index, and body mass index between the aerobic exercise group and the exercise group (*P* > 0.05). And the two groups of subjects in vital capacity, heart function, sit-ups, push-ups, vertical jump, and sitting body flexion test all meet the relevant experimental test requirements and have the experimental preconditions, so they can carry out this experiment.
5. After paired *t*-test with SPSS19.0 analysis software, all indexes of body composition in the aerobic exercise group had significant changes, and the *P* values were less than 0.05. It shows that after 8 weeks of aerobic exercise, the experimenter's body weight, BMI, body fat (%), lean weight, waist-hip ratio, and other indicators have been well improved. In particular, the weight decreased from 85.2 ± 16.26 kg before exercise to 80.6 ± 14.21 kg, and the average weight decreased by 4.6 kg. Body fat (%) decreased from 30.2 ± 2.15 before training to 28.6 ± 3.01, with an average decrease of 1.6 percentage points. The *P* values of these two indexes were less than 0.01, indicating that the improvement effect was very obvious. The specific indicators are shown in Table 5.
6. On the whole, compared with the aerobic exercise group, the resistance exercise group not only has a significant effect on improving body weight and body fat (%) but also has a significant effect on increasing lean body weight. After resistance exercise, the thin weight of the experimenter increased from 54.3 ± 12.23 kg before training to 56.8 ± 10.6 kg. The average increase was about 2.5 kg; *P* value was less than 0.01; and the improvement effect was better.
7. According to the distribution of the population, the changes in body composition indexes in the aerobic exercise group and the exercise group were re-examined and compared. After combining the *t*-test with SPSS19.0 analysis software, the test results are shown in Table 6.

As one of the main indicators of exercise weight loss, weight has always been an important indicator concerned many weight loss participants. We can see from Table 6 that no matter the normal population or the overweight and obese population, there is no significant change in the weight change of the three groups during aerobic exercise and resistance exercise, and the *P* value is greater than 0.05. It shows that there is no significant difference between aerobic exercise and resistance exercise in weight loss and control, and the effects of the two kinds of exercise in improving weight are basically the same.

BMI is translated into Chinese as body mass index, which mainly refers to the corresponding relationship between human height and their own weight. Body mass index has high accuracy and authority in evaluating human body weight. The calculation method mainly calculates the specific value by dividing the self body weight by the square of my height, expressed as kg/m^2^. Relevant studies have pointed out that when the body mass index reaches or exceeds 25 kg/rrf, the body shape is generally obese, and the problems and diseases caused by obesity may be significantly improved [27]. As can be seen from Table 6, there was no significant difference in BMI between normal weight, overweight, and obese people after aerobic exercise or exercise [28]. *P*=0.05. This also shows that aerobic exercise and resistance exercise have basically the same effect on improving the experimenter's body mass index, and the research results are also in line with the changes of body mass index. Lean body weight, also known as fat-free body weight, is one of the important evaluation indicators of body composition and one of the factors concerned by many weight loss and body shaping people, especially male sports lovers. We can clearly see in Figures 8 and 9.

Whether normal people or overweight and obese people, the effect of resistance exercise on increasing lean weight is significantly better than aerobic exercise, *P* < 0.01. This is also closely related to the form and load arrangement of resistance exercise. Resistance movement is the movement of human muscles to actively overcome external resistance, and its effect on increasing muscle content is also very significant.

## 5. Conclusion

Through 8 weeks of exercise, fat reduction, aerobic exercise, and resistance exercise can significantly improve the effect of adult weight loss. Both exercise methods can effectively improve human body composition, enhance cardiopulmonary function, and improve physical quality. Through experimental comparison, aerobic exercise and resistance exercise have little difference in improving body weight, BMI, and waist-hip ratio. People with normal weight can increase their lean weight through aerobic exercise and resistance exercise, but for overweight and obese people, resistance exercise is better than aerobic exercise in reducing fat content. In terms of cardiopulmonary function, the overall improvement effect of aerobic exercise is better than resistance exercise, especially in enhancing the heart function of subjects, which is significantly higher than resistance exercise. Aerobic exercise can effectively improve the heart tolerance and level of participants. Resistance exercise is obviously better than aerobic exercise in improving the level of the body and upper limbs such as sit-ups and push-ups, but aerobic exercise has a better effect in terms of body flexibility such as sitting forward flexion. Aerobic exercise and resistance exercise are helpful to improve the vertical jump strength of lower limbs, but there is no significant difference between them.

## Figures and Tables

**Figure 1:** Wayne diagram of the relationship between deep learning and machine learning.

**Figure 2:** Learning algorithm.

**Figure 3:** Relationship between feature set and training error and generalization error.

**Figure 4:** Single neuron model.

**Figure 5:** Stochastic simulation of regression model 1.

**Figure 6:** Stochastic simulation of regression model 2.

**Figure 7:** Random simulation of the polynomial model.

**Figure 8:** Changes in body fat after aerobic exercise and resistance exercise.

**Figure 9:** Changes in lean body mass index after aerobic exercise and resistance exercise.

**Table 1:** Basic information of research objects.

Gender	Number of people	Age (years)	Height (CM)	Weight (kg)
Male	16	38.10 ± 6.45	173.63 ± 5.98	95.37 ± 10.27
Female	14	36.71 ± 8.28	162.57 ± 5.24	75.95 ± 11.44

**Table 2:** Comparison of test results before intervention.

Group	Weight (kg)	BMI	Body fat (%)	Lean weight (kg)	Waist-hip ratio
Aerobic exercise group	85.2 ± 16.26	27.2 ± 1.16	30.2 ± 2.15	53.1 ± 11.15	1.01 ± 0.08
Resistance exercise group	85.5 ± 15.52	26.4 ± 1.17	29.8 ± 1.88	54.3 ± 12.23	0.99 ± 0.07
Sig	0.98	0.87	0.83	0.74	0.86

*Note.* ^*∗*^ *P* < 0.05 and ^*∗∗*^*P* < 0.01.

**Table 3:** Comparison of cardiopulmonary function results.

Group	Vital capacity (ml)	Cardiac function (MET)
Aerobic exercise group	3,158 ± 288.46	6.7 ± 1.91
Resistance exercise group	3,126 ± 228.35	6.8 ± 2.01
Sig	0.65	0.71

*Note.* ^*∗*^ *P* < 0.05 and ^*∗∗*^*P* < 0.01.

**Table 4:** Comparison of physical fitness results.

Group	Sit-ups	Push-ups (times)	Forward flexion of sitting body (cm)	Vertical jump (cm)
Aerobic exercise group	6.1 ± 3.8	5.5 ± 3.8	1.8 ± 4.3	15.1 ± 4.2
Resistance exercise group	5.8 ± 3.8	5.4 ± 2.6	2.1 ± 3.8	14.8 ± 3.7
Sig	0.58	0.89	0.76	0.68

*Note.* ^*∗*^ *P* < 0.05 and ^*∗∗*^*P* < 0.01.

**Table 5:** Comparison of test results before and after.

Aerobic training experimental group				Resistance training experimental group		
Index	Before training	After training	Sig	Before training	After training	Sig
Weight	85.24 ± 6.26	80.6 ± 14.21	0.00	85.5 ± 15.52	80.5 ± 11.26	0.00
BMI	27.2 ± 1.16	25.2 ± 1.02	0.16	26.4 ± 1.17	24.8 ± 1.14	0.12
Body fat (%)	30.2 ± 2.15	28.6 ± 3.01	0.00	29.8 ± 1.88	26.2 ± 1.15	0.00
Lean weight	53.1 ± 11.15	54.2 ± 10.14	0.38	54.3 ± 12.23	56.8 ± 10.6	0.06
Waist-hip ratio	1.02 ± 0.08	0.98 ± 0.16	0.24	0.99 ± 0.07	0.91 ± 0.12	0.18

**Table 6:** Test results of body composition indexes of normal, overweight, and obese people after two kinds of exercise.

Main indicators	Shape	Aerobic training experimental group	Resistance training experimental group	Sig value
Weight (kg)	Normal	3.2 ± 0.1	3.2 ± 0.15	0.63
	Overweight	5.8 ± 2.12	5.9 ± 2.31	0.78
	Obesity	8.1 ± 1.23	7.9 ± 2.34	0.81
	Normal	1.1 ± 0.01	1.1 ± 0.05	0.96

BMI (kg/m)	Overweight	1.5 ± 0.21	1.5 ± 0.23	0.094
	Obesity	2.3 ± 0.24	2.2 ± 0.18	0.089
	Normal	3.1 ± 1.08	3.12 ± 1.11	0.037

Body fat (%)	Overweight	1.2 ± 0.1	3.4 ± 1.28	0.000
	Obesity	1.5 ± 0.13	3.1 ± 2.1	0.000
	Normal	1.4 ± 0.12	1.5 ± 0.14	0.036

Lean weight (kg)	Overweight	1.15 ± 0.08	2.6 ± 1.23	0.000
	Obesity	1.8 ± 0.16	3.1 ± 1.01	0.000
	Normal	0.11 ± 0.08	0.11 ± 0.06	0.093

Waist-hip ratio	Overweight	0.19 ± 0.06	0.19 ± 0.11	0.087
	Obesity	0.11 ± 0.02	0.12 ± 0.06	0.054

## Data Availability

No data were used to support this study.
